The article "Danlou Tablet May Alleviate Vascular Injury Caused by Chronic Intermittent Hypoxia through Regulating FIH-1, HIF-1, and Angptl4" was published in 2022. Journal: Evid Based Complement Alternat Med.

# Danlou Tablet May Alleviate Vascular Injury Caused by Chronic Intermittent Hypoxia through Regulating FIH-1, HIF-1, and Angptl4

**DOI:** 10.1155/2022/4463108

**Published:** 2022-10-15

**Authors:** Yi Rong, Qian Wu, Jingjing Tang, Zhiguo Liu, Qianyu Lv, Xuejiao Ye, Yu Dong, Yuebo Zhang, Guangxi Li, Shihan Wang

**Affiliations:** ^1^Guang'anmen Hospital, China Academy of Chinese Medical Sciences, Beijing 100053, China; ^2^Department of Cardiovascular Medicine, Mayo Clinic, Rochester, MN 55905, USA; ^3^Department of Pulmonary and Critical Care Medicine, Mayo Clinic, Rochester, MN 55905, USA

## Abstract

**Background:**

Danlou tablet (DLT), the traditional Chinese medicine has been commonly used for dyslipidemia, atherosclerosis, and coronary heart disease. Whether it was effective against vascular injury caused by CIH has remained unknown. The aim of the current study was to observe the effects of DLT on chronic intermittent hypoxia (CIH)-induced vascular injury via regulation of blood lipids and to explore potential mechanisms.

**Methods:**

Sixteen 12-week-old male ApoE^−/−^ mice were randomly divided into four groups. The sham group was exposed to normal room air, whereas the other three groups were exposed to CIH. Mice in the CIH + normal saline (NS) group were gavaged with NS. Mice in the CIH + Angptl4-ab group were intraperitoneally injected with Angptl4-antibody. Mice in the CIH + DLT group were gavaged with DLT. After four weeks of intervention, serum lipid concentrations, and serum lipoprotein lipase (LPL) activity were detected. The changes in atherosclerosis in vascular tissue were detected by hematoxylin and eosin (H&E) staining. Quantitative real-time polymerase chain reaction (qRT-PCR) and Western blot analysis were applied to detect the expression levels of hypoxia-induciblefactor-1 (HIF-1), factor-inhibiting HIF-1 (FIH-1), angiopoietin-like 4 (Angptl4), and LPL in different tissues.

**Results:**

CIH exposure increases serum lipid levels, decreases serum LPL activity, and exacerbates atherosclerosis. Both Angptl4-ab and DLT treatment reversed the changes in lipid concentration, LPL activity, and atherosclerosis caused by CIH. In the epididymal fat pad, CIH exposure decreased the expression of FIH-1 and increased the expression of HIF-1, whereas DLT treatment increased the expression of FIH-1 and LPL and inhibited the expression of HIF-1 and Angptl4. In heart tissue, the expression levels of LPL and Angptl4 were not affected by modeling or treatment.

**Conclusions:**

DLT improved vascular damage by improving the increase in blood lipids induced by CIH, potentially by upregulating FIH-1 and downregulating HIF-1 and Angptl4 in adipose tissue. Therefore, DLT may be a promising agent for the prevention and treatment of CIH-induced vascular injury.

The article "Danlou Tablet May Alleviate Vascular Injury Caused by Chronic Intermittent Hypoxia through Regulating FIH-1, HIF-1, and Angptl4" was published in 2022. Journal: Evid Based Complement Alternat Med.

## 1. Introduction

Obstructive sleep apnea (OSA) is a disorder characterized by breathing cessation, sleep fragmentation, intermittent hypoxia, and hypercapnia caused by repeated narrowing or collapse of the upper airway during sleep [1]. Moderate to severe OSA can increase the risk of vascular injury, vascular outcomes, and all-cause mortality [2]. Common factors of vascular injury include vascular remodeling, inflammation, calcification, and atherosclerosis [3]. Early dyslipidemia impairs endothelial function and causes vascular damage, and its severity is related to the duration and degree of dyslipidemia [4]. The main pathology of OSA is CIH [5], which is recognized as an independent risk factor for dyslipidemia and atherosclerosis [6]. CIH can induce and aggravate arteriosclerosis through inflammation, oxidative stress, insulin resistance, apoptosis, vascular endothelial injury, platelet activation, and neuroendocrine imbalance [6–8]. Dyslipidemia is a major risk factor for atherosclerosis, and atherosclerosis is a major cause of cardiovascular disease [9], which is the leading cause of death worldwide [10]. Thus, early intervention in CIH could treat associated dyslipidemia, thereby delaying the formation of arteriosclerosis and relieving vascular injury.

ApoE^−/−^ mice are widely used to establish experimental models of atherosclerosis [11]. Previous studies have shown that CIH can induce dyslipidemia and atherosclerosis in ApoE^−/−^ mice [12] by inhibiting the expression and activity of LPL and affecting the expression of Angptl4, a potential inhibitor of LPL in adipose tissue but not in heart tissue [13–15]. HIF-1 is a major regulator of hypoxia-induced angiogenesis, which regulates Angptl4 [16, 17]. FIH-1 is an asparaginyl *β*-hydroxylase enzyme that hydroxylates Hypoxia inducible factor 1-alpha (HIF-1*α*), preventing its transcriptional activity and adjusting its posttranslation modification. FIH-1 can reduce the transcriptional activity of proteins by inhibiting the interaction between HIF-1*α* and transcriptional co-activator p300/CBP, thus making people adaptive to hypoxia [18, 19]. HIF-1 can regulate the expression of Angptl4. It promotes Angptl4 expression in uveal melanoma, gastric cancer, osteoporosis, and other diseases [20–22]. In CIH disease models, HIF-1 promotes Angptl4-mediated dyslipidemia and upregulates the expression of Angptl4, which, in turn, inhibits LPL activity and catalytic function, resulting in hyperlipidemia [23].

Currently, medications are the mainstay of treatment for CIH-related AS, and nonpharmacologic treatments are used in addition to pharmaceuticals to treat CIH. Treatment with drugs alone is still under preclinical investigation, and the efficacy is unclear [6]. Traditional Chinese medicine has been widely used for the prevention and treatment of diseases for thousands of years. Danlou tablet (DLT) is a representive traditional Chinese medicine for phlegm and blood stasis (Table 1) [24]. It is commonly used for dyslipidemia, atherosclerosis, and coronary heart disease [8, 25]. Previous studies have shown that DLT has anti-inflammatory and antioxidant effects [26, 27], which may counteract CIH. Furthermore, tanshinone IIA, one of the main ingredients of DLT, decreases HIF-1*α* levels under hypoxic conditions [28]. Both HIF-1 and Angptl4 play important roles in the promotion of dyslipidemia and arteriosclerosis in CIH. Previous studies have shown that Angptl4 is highly expressed in fat but less expressed in the heart and skeletal muscle [29]. However, it is still unknown how DLT functions and its mechanism of action to antiatherosclerosis with a CIH.

The article "Danlou Tablet May Alleviate Vascular Injury Caused by Chronic Intermittent Hypoxia through Regulating FIH-1, HIF-1, and Angptl4" was published in 2022. Journal: Evid Based Complement Alternat Med.

This study aimed to assess the therapeutic effects of DLT on vascular injury caused by CIH and to clarify its potential underlying mechanism with FIH-1, HIF-1, and Angptl4 in the fat and heart tissue of mice.

## 2. Materials and Methods

### 2.1. Reagents and Instruments

We used a commercial preparation of DLT (Batch Number: Z20050244, 0.3 g/tablet) obtained from the Jilin Kangnaier Pharmaceutical Group Co., Ltd. (Jilin, China). The VLDL ELISA kit and LPL ELISA kit were purchased from Nanjing Jiancheng Bioengineering Institute (Jiangsu, China, A111–1, A110–2, A113–2, H249, A067). Anti-HIF-1 and anti-LPL were purchased from Abcam (Zhejiang, China, Ab82832, Ab93898); anti-FIH-1, anti-angptl4, and anti-GAPDH were purchased from affinity (Jiangsu, China, DF7354, DF6751, AF7021). TRIzol was purchased from Aidlab (Beijing, China, 252250AX). RIPA lysate and PMSF were purchased from Beyotime (Shanghai, China, P0013B, ST506). The RevertAid first strand cDNA synthesis kit was purchased from Thermo Fisher Scientific, Inc. (USA, #k1622). Tianyi Huiyuan Gene Technology Co. (Guangdong, China) synthesized the primers for synthesis.

### 2.2. Experimental Animal

Sixteen 12-week-old male C57BL/6J ApoE^−/−^ mice (Batch No. SCXK (Hu) 2018–0004; Shanghai Jiesjie Laboratory Animal Technology Co., LTD) were used in our experiment. All mice were bred in the Animal Experiment Center of Guang'anmen Hospital, China Academy of Chinese Medical Sciences, Beijing, China. The housing conditions were maintained at a room temperature of 22 + 2°C, relative humidity of 55% + 5%, and an illumination time of 07 : 00–19 : 00. After 3 days (d) of adaptive feeding, the mice entered the experimental stage.

The article "Danlou Tablet May Alleviate Vascular Injury Caused by Chronic Intermittent Hypoxia through Regulating FIH-1, HIF-1, and Angptl4" was published in 2022. Journal: Evid Based Complement Alternat Med.

### 2.3. Ethics Statement

All experiments involving animals were in accordance with the guidelines of the Institutional Animal Care and Use Committee and approved by the Ethics Committee of Guang'anmen Hospital, Chinese Academy of Chinese Medical Sciences. The ethics codes were IACUC-GAMH-2022-016-01. All efforts were made to minimize the suffering of animals as much as possible.

### 2.4. Animal Modeling and Grouping

The ApoE^−/−^ mice were initially exposed to CIH or room air (21% O_2_). The CIH protocol consisted of 1-min cycles from normoxia (21% O_2_) to hypoxia (6.5% O_2_) for 12 h/d (09 : 00 to 21 : 00) for 28 d. During the remaining 12 h, all mice were exposed to room air (21% O_2_) [30]. All mice were fed a high fat and cholesterol diet twice a day. Daily intake was restricted: each mouse was fed 13 g/d during the first week and an additional 2 g per week for the following three weeks. During the intermittent hypoxia process, diets were not provided. The animals were randomly divided into four groups (*n* = 4 per group) and treated as follows: (a) mice in the sham group were exposed to room air infusion instead of the CIH protocol; (b) mice in the CIH + normal saline (NS) group were exposed to CIH, then received NS gavage (2 ml/time, 1 time per day for 4 weeks); (c) Mice in the CIH + Angptl4-ab group were exposed to CIH, then, injected with Angptl4 antibody (30 mg/kg) intraperitoneally each week. The intervention lasted for 4 weeks. [31]; (d) mice in the CIH + DLT group were exposed to CIH, and then, received DLT gavage at a dose of 250 mg/kg/d for 4 consecutive weeks.

### 2.5. Tissue and Body Fluid Collection

After four weeks of intervention, the mice were anesthetized with 2% isoflurane. Blood was collected from the orbit 5 h after the last administration and centrifuged at 5 000 rpm for 10 min at 4°C. After collection of blood samples, animals were euthanized by cervical dislocation, then, epididymal fat pad and cardiac tissue specimens were dissected. Serum and tissue samples were frozen at −80°C until used for measurement of biochemical parameters.

### 2.6. Blood Lipid and Activity of LPL Examination

Serum low-density lipoprotein (LDL) and very low-density lipoprotein (VLDL) cholesterol levels were detected by an enzyme-linked immunosorbent assay according to the manufacturer's instructions. Activity of LPL was detected using a LPL ELISA Kit according to the manufacturer's instructions.

### 2.7. RNA Extraction and qRT-PCR

Tissue stored in liquid nitrogen was ground and added to Trizol reagent for RNA extraction. cDNA was synthesized using a RevertAid First Strand cDNA Synthesis Kit. qRT-PCR was performed using the Sybr Green experimental method with a fluorescent qRT-PCR instrument (ABI QuantStudio 6). Using the comparison CT value (Δ Δ CT) and GAPDH standardized method to test relative expression of genes in epididymal fat pad and heart tissue. The expression levels of FIH-1, Angptl4, HIF-1, and LPL genes in each group were compared. A dissolution curve was drawn, and final data were analysed with the 2−△△Ct method. The primer sequences used are shown in Table 2.

The article "Danlou Tablet May Alleviate Vascular Injury Caused by Chronic Intermittent Hypoxia through Regulating FIH-1, HIF-1, and Angptl4" was published in 2022. Journal: Evid Based Complement Alternat Med.

### 2.8. Western Blot Analysis

Animal tissues were lysed with RIPA lysate. The protein samples were separated by sodium dodecyl sulfate-polyacrylamide gel electrophoresis (SDS-PAGE) using a Mini-PROTEAN Tetra system (Bio-Rad) and then transferred to polyvinylidene fluoride membranes. Afterward, membranes were blocked using 5% fat-free milk dissolved in Tris Buffered Saline Tween (TBST) for 2 h at room temperature, and then, incubated with primary antibodies against target proteins (FIH-1 : Affinity Inc., DF7354, primary antibody dilution ratio 1 : 500, Angptl4: Affinity Inc., DF6751, primary dilution ratio 1 : 1 000. LPL : Abcam Co., Ltd., Ab93898, primary antibody dilution ratio 1 : 500. HIF-1 : Abcam Co., Ltd., Ab82832, primary antibody dilution ratio 1 : 1 000) at 4°C with gentle shaking overnight. After washing three times with TBST, the membranes were further incubated with secondary antibody (dilution ratio of 1 : 500) at room temperature for 1–2 h. After the reaction, the membranes were washed three times with TBST, and an enhanced chemiluminescence reagent was mixed with stable peroxidase solution at a 1 : 1 ratio. The working solution was then added to the polyvinylidene fluoride membranes and developed the imaging system.

### 2.9. Hematoxylin and Eosin (H&E)

For H&E staining, the fresh isolated tissues were fixed in 4% paraformaldehyde solution for 24–48 h, embedded in paraffin, then cut to 6 *μ*m and mounted on glass slides. The slides were counterstained by hematoxylin (4 min), rinsed with water until slide runs clear. Tissues were dehydrated sequentially with 70, 95 and 100% ethanol, immersed in xylene and cover-slipped using a mounting medium, and images were captured using a panoramic MIDI system from 3DHISTECH.

## 3. Statistical Analysis

Data are presented as the mean ± SD of at least 3 biological replicates. One-way analysis of variance and post hoc Tukey's test were applied to compare the quantitative variables and to analyze the differences among all groups. All statistical tests were performed using IBM SPSS Statistics (v23.0, USA). *P* values of <0.05 and < 0.01 were considered significant and highly significant, respectively.

The article "Danlou Tablet May Alleviate Vascular Injury Caused by Chronic Intermittent Hypoxia through Regulating FIH-1, HIF-1, and Angptl4" was published in 2022. Journal: Evid Based Complement Alternat Med.

## 4. Results

### 4.1. DLT Alleviated Abnormal Changes in Serum Lipid Concentrations and LPL Caused by CIH

We first tested the effects of CIH, Angptl4 antibody, and DLT treatment on serum LDL (Figure 1(a)), VLDL (Figure 1(b)) and LPL (Figure 1(c)) in mice. Compared with the Sham group, CIH treatment significantly increased LDL and VLDL concentrations, but this effect was reduced by Angptl4-ab and DLT treatment (Figures 1(a) and 1(b)). In addition, LPL activity decreased significantly in the CIH group (CIH vs. Sham, *P* < 0.01, Figure 1(c)), whereas Angptl4-ab and DLT treatment increased LPL activity (Figure 1(c)). No significant differences were reported between the DLT and Angptl4-ab groups (Figure 1(c)). Therefore, we concluded that CIH aggravates dyslipidemia, but DLT alleviated this interference and exerted a similar effect as that of Angptl4-ab.

In addition, HE staining was performed on vascular tissues to observe the changes of atherosclerosis. The results showed that the area of atherosclerotic plaque, arterial wall thickening, and lumen narrowing were significantly increased in the sham operation group. Compared with the CIH group, the atherosclerotic plaque areas were significantly reduced in the Angptl4-ab and DLT groups. The artery wall thickness was somewhat narrowed (Figure 1(d)). These results indicate that the atherosclerotic lesion symptoms were significantly induced by CIH, but DLT alleviated this induction and exerted a similar effect as that of Angptl4-ab.

### 4.2. Molecular Mechanism of DLT Improved Vascular Damage Induced by CIH

We tested mRNA expression levels in FIH-1, HIF-1, Angptl4, and LPL in the epididymal fat pads of ApoE^−/−^ mice. Based on qRT-PCR, CIH exposure decreased mRNA expression of FIH-1 (Figure 2(a)) but increased the expression of HIF-1 and Angptl4 (Figures 2(b) and 2(c)), and did not affect the expression of LPL mRNA. We also showed via Western blot that hypoxia reduced the expression of FIH-1 and increased the Angptl4 and HIF-1 protein level (Figure 3(b), 3(c), and 3(e)). The expression level of LPL was not altered (Figure 3(d)), but this did not conflict with previous study that Angptl4 may only suppress the activity of LPL [14]. These results indicate the involvement of FIH-1, HIF-1, and Angptl4 in CIH-induced dyslipidemia.

Both FIH-1 and LPL were markedly upregulated in the DLT group, whereas HIF-1 and Angptl4 were downregulated (Figures 3(b) and 3(c)). Thus, DLT may exert a protective role in lipid metabolism by antagonizing the regulating effect of hypoxia on FIH-1, HIF-1, and Angptl4.

In heart tissue, CIH exposure resulted in decreased expression of FIH-1 mRNA (Figures 4(a)), increased expression of HIF-1 mRNA (Figure 4(c)), and no change in the expression of Angptl4 or LPL mRNA (Figures 4(b) and 4(d)). Compared with the CIH group, the expression of FIH-1 and HIF-1 mRNA in the DLT group was significantly increased (Figure 4(a)) and significantly decreased (Figure 4(c)), respectively. However, no changes in the expression of Angptl4 and LPL mRNA (Figures 4(b) and 4(d)) were observed. The Western blot results revealed that the Angptl4 and LPL protein levels showed a nonsignificant increase (Figures 5(c) and 5(d)). The HIF-1 protein level was upregulated under a CIH exposure, and the FIH-1 protein level decreased. In contrast, Angptl4-ab and DLT reversed this change (Figures 5(b) and 5(e)).

The article "Danlou Tablet May Alleviate Vascular Injury Caused by Chronic Intermittent Hypoxia through Regulating FIH-1, HIF-1, and Angptl4" was published in 2022. Journal: Evid Based Complement Alternat Med.

## 5. Discussion

CIH is a vital pathological characteristic of OSA, which is closely related to lipid metabolism abnormities, eventually leading to atherosclerosis and other metabolic related diseases. A meta-analysis showed that patients after surgeries for OSA had lower blood lipids and the degree of OSA improvement was positively correlated with the improvement of lipid profile parameters [32]. DLT has been proved to be effective in lowering blood lipids and antiatherosclerosis through a variety of mechanisms, including activating PI3K/Akt/mTOR-mediated autophagy of vascular adventitial fibroblasts [33], inhibiting of the NF-*κ*B-mediated inflammatory response [34], and attenuating macrophage foam cell formation via the TLR4/NF-*κ*B and PPAR*γ* signaling pathways [35]. In the current study, we found that CIH exposure aggravated dyslipidemia in ApoE^−/−^ mice, but that DLT treatment effectively improved the dyslipidemia and alleviated the decrease in LPL activity caused by hypoxia. The underlying mechanism related to the effects of DLT on CIH-induced dyslipidemia may be associated with the upregulation of FIH-1 and downregulation of HIF-1 and Angptl4. Our results suggest that DLT may be a promising agent for dyslipidemia treatment in CIH patients. Thus, DLT may play a role in improving vascular injury by reducing dyslipidemia caused by CIH.

Angptl4, a member of the Angptl4 family, is expressed in both humans and mice. It can effectively inhibit LPL activity, affect lipid metabolism, delay triglyceride clearance in the blood, and finally, lead to increased blood lipids and arteriosclerosis [36]. The human Angptl4 E40K mutation can deactivate Angptl4, thereby reducing triglycerides, increasing high-density lipoprotein cholesterol, and reducing dyslipidemia and arteriosclerosis [37], as well as the incidence of cardiovascular disease [38]. The monoclonal antibody injected with human Angptl4 in mice and monkeys can also inhibit triglyceride levels and improve atherosclerosis and dyslipidemia [30, 31, 36, 37]. Therefore, research on the treatment of dyslipidemia and atherosclerosis with angiopoietin-like 3 and Angptl4-related antibodies has also emerged [39], although such treatment has not yet been widely used in clinical practice.

The article "Danlou Tablet May Alleviate Vascular Injury Caused by Chronic Intermittent Hypoxia through Regulating FIH-1, HIF-1, and Angptl4" was published in 2022. Journal: Evid Based Complement Alternat Med.

As the main regulator of Angptl4 [40, 41], HIF-1 plays a role in promoting arteriosclerosis and dyslipidemia by upregulating Angptl4, inhibiting the expression of LPL, and increasing triglycerides and lipids in CIH-induced lipid metabolism and arteriosclerosis [14]. We also found an increase in the levels of HIF-1, Angptl4, and lipid profiles in the epididymal fat tissue of CIH-exposed mice, confirming the role of HIF-1 in regulating lipid profiles under CIH conditions.

Notably, in heart tissue, although HIF-1 was increased in the CIH group, no differences in Angptl4 were observed among the groups, which may be related to the different expression levels of Angptl4 in each tissue [40, 41]. Our study suggests that the HIF-1-Angptl4 pathway may work through adipose tissue [14].

FIH-1 is an asparagine-basedbeta-hydroxylase that inhibits HIF-1*α* transcriptional activity, and regulates fat metabolism and affects insulin sensitivity [42]. Previous studies have shown that inhibiting HIF-1 could result in renal protection [43], tumor angiogenesis [44], and hypoxia response of tumor cells [45]. However, few studies have examined the impact of FIH-1 on lipid metabolism [46]. We assumed that FIH-1 may be involved in lipid metabolism under hypoxic conditions through regulating HIF-1 and Angptl4. Here, qRT-PCR and Western blot analysis of epididymal fat tissue samples indicated that CIH exposure resulted in decreased expression of FIH-1 and LPL and increased expression of HIF-1 and Angptl4. Of note, administration of DLT reversed these changes, with a significantly lower lipid profile and an increased level of LPL. DLT also regulates FIH-1, HIF-1, and Angptl4 in the meantime. Therefore, FIH-1, HIF-1, and Angptl4 may play important roles in the treatment of dyslipidemia caused by CIH.

In heart tissue, CIH exposure led to decreased expression of FIH-1, increased expression of HIF-1, but no change in the expression of Angptl4 or LPL. In addition, in the intervention groups, the expression levels of FIH-1 were significantly increased by Angptl4 antibody and DLT treatment, which inhibited the expression of HIF-1 but had no significant effect on the expression levels of Angptl4 and LPL, which may be explained by possible multiple upstream regulators of Angptl4 [47].

Hyperlipidemia is closely related to vascular injury, which can start in childhood and worsen with age [48]. Dyslipidemia usually causes vascular injury through inflammation, immune response, and oxidative stress [49]. CIH can lead to hyperlipidemia, which can further damage blood vessels [50]. Therefore, intervening in dyslipidemia induced by CIH could alleviate inflammation and improve lipid metabolism and blood vessel damage. Our study indicated that DLT treatment may alleviate CIH-induced dyslipidemia, and thus, may also reduce vascular damage caused by CIH.

The article "Danlou Tablet May Alleviate Vascular Injury Caused by Chronic Intermittent Hypoxia through Regulating FIH-1, HIF-1, and Angptl4" was published in 2022. Journal: Evid Based Complement Alternat Med.

In our study, indicated that the serum concentrations of LDL, VLDL, and LPL in CIH-exposed mice were reduced by DLT treatment; we also demonstrated that this treatment could reduce serum total cholesterol (TC) and triglyceride (TG) levels in a previous study [8]. After DLT intervention, by regulating FIH-1, HIF-1, and Angptl4, the expression level of LPL increased significantly. Therefore, our results suggest that DLT upregulates FIH-1 and downregulates HIF-1 and Angptl4 in adipose tissue, thereby reducing CIH-induced vascular injury.

This study has some limitations. First, previous studies have indicated that FIH-1 Adenosine Monophosphate Activated Protein Kinase and Proliferator-activatedreceptor-gamma coactivator 1-alpha factors can also regulate HIF-1 [51, 52], which can affect lipid metabolism. In lipid metabolism, HIF-1 can regulate lipids via the SREBP-1 pathway [53]. Therefore, the interaction between molecular substances in signaling pathways and other signaling pathways should be fully considered. Second, further cellular experiments are needed to verify the targeted regulation of HIF-1*α* by DLT. This is complemented by our previously cell experiment which proved DLT had positive effects in improving dyslipidemia and arteriosclerosis by inhibiting Angptl4 protein levels through HIF-1*α*-Angptl4 mRNA signaling pathway. In addition, as a compound preparation, many single ingredients of DLT have been demonstrated to be effective against dyslipidemia [54–56]; however, the effects of the compound still need to be further studied with more drug metabolomics research, which is our future direction of study.

## 6. Conclusions

DLT improved vascular damage by improving the increase in blood lipids induced by CIH, potentially via upregulating FIH-1 and downregulating HIF-1 and Angptl4 in adipose. Thus, DLT may be a promising agent for the prevention and treatment of CIH-induced vascular injury.

## Figures and Tables

**Figure 1:** Determination of serum lipids, lipoproteins and H&E staining. (a) serum LDL of ApoE^−/−^ mice in each group; (b) serum VLDL of ApoE^−/−^ mice in each group; (c) serum LPL activity of ELISA of ApoE^−/−^ mice in each group; (d) Representative images of haematoxylin and eosin staining of ApoE^−/−^ mice in each group. Bar = 50 *μ*m. One-way analysis of variance and post hoc Tukey's test was applied to compare the lipids and lipoproteins and to analyze the difference among all groups. ^*∗∗*^*P* < 0.01 (vs. Sham);  ^*∗*^*P* < 0.05 (vs. Sham); ^##^*P* < 0.01 (vs. CIH); ^#^*P* < 0.05 (vs. CIH).

The article "Danlou Tablet May Alleviate Vascular Injury Caused by Chronic Intermittent Hypoxia through Regulating FIH-1, HIF-1, and Angptl4" was published in 2022. Journal: Evid Based Complement Alternat Med.

**Figure 2:** qRT-PCR analysis of epididymal fat pad of ApoE^−/−^ mice in each group. (a) FIH-1 mRNA expression level; (b) Angptl4 mRNA expression level; (c) HIF-1 mRNA expression level; (d) LPL mRNA expression level. One-way analysis of variance and post hoc Tukey's test was applied to compare the qRT-PCR analysis of epididymal fat pad and to analyze the difference among all groups. ^*∗∗*^*P* < 0.01 (vs. Sham),  ^*∗*^*P* < 0.05 (vs. Sham); ^##^*P* < 0.01 (vs. CIH); ^#^*P* < 0.05 (vs. CIH).

**Figure 3:** Western blot analysis of epididymal fat pad of ApoE^−/−^ mice in each group. (a) cropped blots; (b) FIH-1 protein level; (c) Angptl4 protein level; (d) LPL protein level; (e) HIF-1 protein level. One-way analysis of variance and post hoc Tukey's test was applied to compare the Western blot analysis of epididymal fat pad and to analyze the difference among all groups. ^*∗∗*^*P* < 0.01 (vs. Sham); ^*∗*^*P* < 0.05 (vs. Sham); ^##^*P* < 0.01 (vs. CIH); ^#^*P* < 0.05 (vs. CIH).

**Figure 4:** qRT-PCR analysis of heart tissues of ApoE^−/−^ mice in each group. (a) FIH-1 mRNA expression level; (b) Angptl4 mRNA expression level; (c) HIF-1 mRNA expression level; (d) LPL mRNA expression level. One-way analysis of variance and post hoc Tukey's test was applied to compare the qRT-PCR analysis of heart tissues and to analyze the difference among all groups. ^*∗∗*^*P* < 0.01 (vs. Sham);  ^*∗*^*P* < 0.05 (vs. Sham); ^##^*P* < 0.01 (vs. CIH); ^#^*P* < 0.05 (vs. CIH).

**Figure 5:** Western blot analysis of heart tissue of ApoE^−/−^ mice in each group: (a) Cropped blots; (b) FIH-1 protein level; (c) Angptl4 protein level; (d) LPL protein level; (e) HIF-1 protein level. One-way analysis of variance and post hoc Tukey's test was applied to compare the Western blot analysis of heart tissueand to analyze the difference among all groups. ^*∗∗*^*P* < 0.01 (vs. Sham);  ^*∗*^*P* < 0.05 (vs. Sham); ^##^*P* < 0.01 (vs. CIH); ^#^*P* < 0.05 (vs. CIH).

**Table 1:** Scientific species names of all ingredients of the Danlou tablet.

Chinese name	English name	Latin name	Amount (g)	Percentage of ingredient (%)
*Gualou*	*Fructus trichosanthis*	*Fructus trichosanthis kirlowii*	86	10.20
*Danshen*	*Danshen root*	*Radix salviae miltiorrhizae*	138	16.51
*Xiebai*	*Bulbus allii macrostemonis*	*Bulbus allii*	40	4.78
*Chuanxiong*	*Rhizoma chuanxiong*	*Radix ligustici wallichii*	52	6.22
*Chishao*	*Radix paeoniae rubra*	*Radix rubrus paeoniae lactiflorae*	52	6.22
*Yujin*	*Radix Curcumae*	*Tuber curcumae*	52	6.22
*Huangqi*	*Radix astragali*	*Radix astragali membranacei*	114	13.64
*Gegen*	*Radix puerariae*	*Radix puerariae*	138	16.51
*Zexie*	*Rhizoma alismatis*	*Rhizoma alismatis*	138	16.51
*Gusuibu*	*Radix dryariae*	*Radix dryariae*	26	3.11

The article "Danlou Tablet May Alleviate Vascular Injury Caused by Chronic Intermittent Hypoxia through Regulating FIH-1, HIF-1, and Angptl4" was published in 2022. Journal: Evid Based Complement Alternat Med.

**Table 2:** Primer sequence.

The name of the primer	Primer sequence (5′-3′)	Fragment length (bp)
mFIH-1-F	GTCCCAGCTACGAAGTTACAGC	136
mFIH-1-R	CAGTGCAGGATACACAAGGTTT	
mAngptl4-F	CATCCTGGGACGAGATGAACT	136
mAngptl4-R	TGACAAGCGTTACCACAGGC	
mLPL-F	TTGCCCTAAGGACCCCTGAA	88
mLPL-R	TTGAAGTGGCAGTTAGACACAG	
mHIF-1a-F	TCTCGGCGAAGCAAAGAGTC	214
mHIF-1a-R	AGCCATCTAGGGCTTTCAGATAA	
GAPDH-mF	AAGGCTGTGGGCAAGG	238
GAPDH-mR	TGGAGGAGTGGGTGTCG	
mHIF-1aF	TCTCGGCGAAGCAAAGAGTC	214
mHIF-1aR	AGCCATCTAGGGCTTTCAGATAA	

## Data Availability

The datasets used and/or analysed during the current study are available from the corresponding author on reasonable request.

## Abbreviations

Angptl4: Angiopoietin-like 4
CIH: Chronic intermittent hypoxia
DLT: Danlou tablet
FIH: Factor-inhibiting HIF-1
HIF-1: Hypoxia-inducible factor-1
HIF-1*α*: Hypoxia inducible factor 1-alpha
LDL: Low density lipoprotein
LPL: Lipoprotein lipase
NS: Normal saline
OSA: Obstructive sleep apnea
qRT-PCR: Quantitative real-time polymerase chain reaction
TBST: Tris buffered saline tween
TC: Total cholesterol
TG: Triglyceride
VLDL: Very low-density lipoprotein cholesterol.
